The article "Automatic Target Recognition of SAR Images Using Collaborative Representation" was retracted in 2023. Reasons: signs of a paper mill; compromised peer review; unreliable results or conclusions.

# Automatic Target Recognition of SAR Images Using Collaborative Representation

**DOI:** 10.1155/2022/3100028

**Published:** 2022-05-24

**Authors:** Jinge Hu

**Affiliations:** Chongqing Three Gorges University, Chongqing 404100, China

## Abstract

Synthetic aperture radar (SAR) automatic target recognition (ATR) is one of the key technologies for SAR image interpretation. This paper proposes a SAR target recognition method based on collaborative representation-based classification (CRC). The collaborative coding adopts the global dictionary constructed by training samples of all categories to optimally reconstruct the test samples and determines the target category according to the reconstruction error of each category. Compared with the sparse representation methods, the collaborative representation strategy can improve the representation ability of a small number of training samples for test samples. For SAR target recognition, the resources of training samples are very limited. Therefore, the collaborative representation is more suitable. Based on the MSTAR dataset, the experiments are carried out under a variety of conditions and the proposed method is compared with other classifiers. Experimental results show that the proposed method can achieve superior recognition performance under the standard operating condition (SOC), configuration variances, depression angle variances, and a small number of training samples, which proves its effectiveness.

## 1. Introduction

Synthetic aperture radar (SAR) can work continuously under all-weather conditions, thus providing an effective tool for intelligence reconnaissance. SAR automatic target recognition (ATR), as an important research content of SAR image interpretation [1], has been extensively studied in the past 20 years. Specific SAR target recognition methods mainly focus on two technologies: feature extraction and classifier design. Feature extraction aims to reduce the dimensionality of the original SAR data, thereby facilitating the subsequent decision making. The features commonly used in SAR target recognition include target region, target contour [2–7], scattering centers [8–10], principal component analysis (PCA) features, linear discriminant analysis (LDA) features, image decompositions [11–18], etc. The classifier design aims to make decisions on the original SAR image or the extracted features to determine the target category. With the advancement of pattern recognition technology, a large number of classifiers have been applied in SAR target recognition, such as K-nearest neighbor (KNN) [8], support vector machine (SVM) [19–21], sparse representation-based classification (SRC) [22–27], convolutional neural network (CNN) [28–39], and so on. Mishra applied PCA and LDA to SAR image feature extraction and classified them through KNN [11]. The authors in [2] first extracted the elliptical Fourier descriptor of the SAR target contour and then used the SVM classifier for target recognition. In [8], the authors proposed an attribute scattering center matching algorithm and applied it to SAR target recognition. The authors in [19, 23] applied SVM and SRC to SAR target recognition, respectively, and proved their effectiveness. The scope of application and classification performance of different classifiers are usually not the same. Therefore, in order to improve the recognition performance, it is necessary to select a more effective and robust classifier.

The article "Automatic Target Recognition of SAR Images Using Collaborative Representation" was retracted in 2023. Reasons: signs of a paper mill; compromised peer review; unreliable results or conclusions.

In this paper, the collaborative representation-based classification (CRC) [40–42] is applied to SAR target recognition. The basic idea is to use a global dictionary composed of various training samples to optimally reconstruct test samples and then determine the target category according to various reconstruction errors. Zhang et al. [40] first proposed a collaborative representation classifier and applied it to face recognition with good results. The results also proved that under the condition of limited training samples in each category, the strategy of using collaborative representation is more robust than the traditional sparse representation. For SAR target recognition, limited by the ability to acquire data, the number of training samples in each category is often very limited, so it is more appropriate to use collaborative representation during the classification. In order to scientifically test the proposed method, the moving and stationary target acquisition and recognition (MSTAR) dataset is used to conduct verification experiments under different conditions, and the superiority of the proposed method is verified by comparison with other classifiers.

## 2. SRC

Sparse representation is essentially a linear representation theory [22–27]. Different from the general linear representation, the sparse representation requires the linear representation coefficients to be sparse, that is, only a small number of coefficients are nonzero. Suppose that the global dictionary constructed by *C* classes of targets is *A*=[*A*^1^, *A*^2^,…, *A*^*C*^] ∈ *R*^*d*×*N*^, where *d* is the dimension of each atom (i.e., the feature vector extracted from the training sample) and *A*^*i*^ ∈ *R*^*d*×*N*_*i*_^(*i*=1,2,…, *C*) denotes the *N*_*i*_ atoms from the *i*th class. For the test sample *y* ∈ *R*^*d*^, the following equation is used for sparse representation:

(1) $$\begin{array}{c} \hat{\alpha }=\arg\min{\left\|\alpha \right\|}_{0}\;s.t.{\left\|y-A\alpha \right\|}_{2}^{2}\leq \varepsilon . \end{array}$$

In (1), *α* represents the sparse representation coefficient vector and *ε* is the reconstruction error. The above problem is difficult to be directly solved because it involves the *ℓ*_0_ norm optimization. According to the research results of compressive sensing theory, the *ℓ*_1_ minimization algorithm, orthogonal matching pursuit (OMP), Bayesian compressive sensing (BCS), etc. can be used to obtain the approximate solution of problem (1).

The article "Automatic Target Recognition of SAR Images Using Collaborative Representation" was retracted in 2023. Reasons: signs of a paper mill; compromised peer review; unreliable results or conclusions.

On the basis of obtaining the sparse representation coefficient vector $\hat{\alpha }$, the target category is determined by calculating the reconstruction error of each training category with regard to the test sample, as shown below:

(2) $$\begin{array}{c} r\left(i\right)={\left\|y-A_{i}{\hat{\alpha }}_{i}\right\|}_{2}^{2}\left(i=1,2,\ldots ,C\right),\\ \text{identity}\left(y\right)=\underset{i}{\arg\min}\left(r\left(i\right)\right). \end{array}$$

In (2), ${\hat{\alpha }}_{i}$ represents the partial coefficients corresponding to the *i*th class and *r*(*i*)(*i*=1,2,…, *C*) is the reconstruction error of each training class to the test sample. Finally, the test sample is determined as the category that obtains the smallest reconstruction error.

## 3. CRC

The sparse representation in SRC emphasizes the effect of sparsity on target recognition but ignores the complementarity of different categories. When the number of training samples of each category in the dictionary is limited, it is difficult to achieve a high-precision description of the test samples by using sparse representation. In this situation, the classification results based on sparse representation may bring false judgments. Collaborative representation means that the joint use of samples of different types can provide a more accurate description of the test samples. Therefore, CRC uses the least regularized mean square error algorithm to solve the collaborative coding coefficients on the global dictionary as follows [39]:

(3) $$\begin{array}{c} \hat{x}=\arg\min\left\{{\left\|y-Ax\right\|}_{2}^{2}+\lambda {\left\|x\right\|}_{2}^{2}\right\}. \end{array}$$

In (3), *λ* is the regularization coefficient. Compared with the sparse representation coefficients, the solution of cooperative coding is much simpler. The analytical solution of (3) can be calculated as follows:

(4) $$\begin{array}{c} \hat{x}={\left(A^{T}A+\lambda *I\right)}^{-1}A^{T}y. \end{array}$$

In (4), *I* is an identity matrix. According to the solved collaborative representation coefficient, using the same method as (2), the reconstruction error of each category is calculated and the target category is judged based on the smallest representation error. Compared with SRC, the collaborative representation strategy can better characterize the test samples. In addition, the *ℓ*_2_ norm minimization in (3) is a convex optimization algorithm, which is simpler and more efficient than the *ℓ*_0_ norm optimization in (1).

The article "Automatic Target Recognition of SAR Images Using Collaborative Representation" was retracted in 2023. Reasons: signs of a paper mill; compromised peer review; unreliable results or conclusions.

This paper applies CRC to SAR target recognition, and its specific implementation is described as follows. In order to reduce the dimensionality of the original SAR data, PCA is used for feature extraction. The PCA features of the training samples are used to construct a global dictionary, and then the PCA feature of the test sample is collaborative represented based on the global dictionary. Finally, the target category is determined according to the resulting reconstruction errors.

## 4. Experiments

### 4.1. Description of Dataset

In order to verify the recognition performance of the method in this paper, the experiments are carried out on the MSTAR dataset. The dataset collects the measured SAR images of 10 types of ground stationary targets by the X-band sensors, which were published by the US DARPA/AFRL. The image resolution is 0.3 m × 0.3 m, which is an important dataset for testing SAR target recognition methods.  Figure 1 shows some examples of the optical and SAR images of 10 types of targets.  Table 1 lists the training and test samples used in this paper. In the experiment, 10 types of target images at the depression angle of 17° are used as training samples, and 10 types of target images at the depression angle of 15° are used as the test samples to be recognized.

### 4.2. Results and Discussion

In order to fully verify the effectiveness of the method in this paper, the CRC is compared with several classic SAR target recognition classifiers, including the KNN, SVM, SRC, and CNN. In order to ensure the consistency of the comparison, the classifiers KNN, SVM, and SRC also classify the extracted PCA feature vectors like CRC. All methods are run based on MATLAB 2016, and the hardware platform is a personal computer with a 3.4 GHz Intel i7 processor and 8G memory.

#### 4.2.1. 10-Class Recognition

First, the test samples of 10 types of targets in Table 1 are classified based on the training samples. The recognition results of the method in this paper are shown in Figure 2. It can be seen that the CRC method proposed in this paper has an average recognition rate of 96.92% for 10 types of targets, which fully demonstrates its effectiveness.  Table 2 compares the average recognition rates and time consumption of CRC and other types of SAR target recognition methods for 10 types of targets. The method in this paper has the highest recognition rate, which shows the high performance of the proposed method. By comparing the CRC and SRC methods, it can be seen that the collaborative representation strategy adopted by CRC effectively improves the target recognition performance compared to the sparse representation algorithm. Comparing the time consumption of various methods to recognize a single MSTAR image under the same hardware platform, the proposed method has higher efficiency. As shown in (4), the CRC solution can be smoothly obtained using the convex optimization. Therefore, it can achieve much higher efficiency. The performance of the CNN method ranks second under this condition mainly because of the high classification capability of deep learning when the training samples are sufficient to cover the test samples.

The article "Automatic Target Recognition of SAR Images Using Collaborative Representation" was retracted in 2023. Reasons: signs of a paper mill; compromised peer review; unreliable results or conclusions.

#### 4.2.2. Performance at Different Feature Dimensions

The performance of the classifier is closely related to the extracted features. In order to further test the recognition robustness of the CRC method, this paper conducts recognition experiments on 10 types of targets in different feature dimensions.  Table 3 shows the performance curves of the KNN, SVM, and SRC methods as the PCA feature dimensions change. All these methods maintain a relatively close recognition performance within a given feature dimension. In contrast, the CRC method proposed in this paper has the highest average recognition rate in each dimension, which proves its superiority. The CNN method is not compared in this condition because the deep networks are directly trained based on the image intensities rather than the extracted PCA feature vectors.

#### 4.2.3. Configuration Variance

Configuration variances are more common in military targets. For example, a certain type of tank can be transformed into another configuration through local structural adjustments. This type of difference will have a certain impact on target recognition performance. In order to test the recognition performance of the CRC method under configuration variances, part of the training and test samples in Table 1 is used to perform recognition experiments, as shown in Table 4. Among them, the training and test samples of BMP2 and T72 targets have some configuration differences.  Table 5 lists the recognition performance of various methods under configuration variances. Compared with the average recognition rates under the 10-class recognition condition in Table 2, the performance of various methods under the condition of configuration variances has declined to varying degrees. In contrast, the CRC method proposed in this paper achieves the highest recognition performance under configuration variances, reflecting its effectiveness for configuration changes. Collaborative representation has stronger representation ability for test samples with different configurations, thereby improving the performance of target recognition.

The article "Automatic Target Recognition of SAR Images Using Collaborative Representation" was retracted in 2023. Reasons: signs of a paper mill; compromised peer review; unreliable results or conclusions.

#### 4.2.4. Depression Angle Variance

The difference in the depression angle will cause the acquired SAR image to undergo a large change. At this time, the performance of target recognition tends to be severely degraded.  Table 6 shows the training and test samples used in this experiment. There is a big difference in depression angle between the training and the test sets. The recognition performance of various algorithms is shown in Table 7. When the change in depression angle is relatively small (e.g., from 17° to 30°), various methods can still have higher recognition rates. When the depression angle changes greatly (e.g., from 17° to 45°), the recognition performance of various algorithms has experienced a sharp drop. In contrast, the CRC method proposed in this paper maintains the highest average recognition rates at both 30° and 45° depression angles, which proves that it has strong robustness to depression angle changes. Similar to the case of configuration variances, the collaborative representation has good capability to represent the test samples with large depression angle differences. Therefore, the CRC method proposed in this paper could achieve better robustness to possible depression angle variances.

#### 4.2.5. Few Training Samples

Limited by the ability of SAR data acquisition, the training samples available in the actual process are very limited compared to the large number of samples to be identified. Therefore, the stability of the recognition algorithm under a small number of training samples is very critical. In order to test the robustness of the CRC method under a small number of training samples, this paper takes 20%, 40%, 60%, and 80% of the original training samples in Table 1 to form the training set and then test the recognition performance of different methods. The performance comparison of various methods is shown in Figure 3. It can be seen that with the reduction of training samples, the recognition performance of various methods has been significantly reduced. In contrast, the CRC method is least affected by the reduction of training samples and maintains the highest average recognition rates on the training sets of various sizes. Therefore, the collaborative representation strategy adopted by CRC effectively improves the recognition performance of the proposed method under a small number of training samples.

## 5. Conclusion

This paper proposes a SAR target recognition method based on CRC. Compared with the traditional sparse representation, the collaborative representation strategy can comprehensively utilize various training samples to achieve higher-precision representations of the test samples, thereby improving the ability to represent the test samples under the condition of a small number of training samples. The CRC is applied to SAR target recognition, and experimental verification is carried out on the MSTAR dataset. The results show that the method in this paper has a recognition rate of 96.92% for 10 types of MSTAR targets, which shows its good performance. Through testing the recognition performance under different feature dimensions, configuration variances, depression angle variances, and a small number of training samples, the results further show the robustness of the CRC method to different kinds of extended operating conditions. All these illustrate the superiority of the method in this paper and prove that it has great application potential in SAR target recognition.

The article "Automatic Target Recognition of SAR Images Using Collaborative Representation" was retracted in 2023. Reasons: signs of a paper mill; compromised peer review; unreliable results or conclusions.

## Figures and Tables

**Figure 1:** Optical and SAR images of the targets in the MSTAR dataset. (a) BMP2, (b) BTR70, (c) T72, (d) T62, (e) BRDM2, (f) BTR60, (g) ZSU23/4, (h) D7, (i) ZIL131, (j) 2S1.

**Figure 2:** The recognition results of 10 classes of targets.

**Figure 3:** Comparison of results under few training samples.

**Table 1:** Training and test samples used in this paper.

Type	BMP2	BTR70	T72	T62	BDRM2	BTR60	ZSU23/4	D7	ZIL131	2S1
Training set	233 (Sn_9563)	233	232 (Sn_132)	299	298	256	299	299	299	299

Test set	195 (Sn_9563)	196	196 (Sn_132)	273	274	195	274	274	274	274
	196 (Sn_9566)		195 (Sn_812)							
	196 (Sn_c21)		191 (Sn_s7)							

**Table 2:** Performances of different methods on 10 classes of targets.

Method type	CRC	KNN	SRC	SVM	CNN
Average recognition rate (%)	97.22	94.35	95.64	95.82	96.04
Time consumption (ms)	25.3	40.3	32.1	24.6	36.23

**Table 3:** The recognition performances of different methods at different feature dimensions.

Feature dimension	40	60	80	100	120
Average recognition rate (%)	95.23	96.02	96.92	96.38	96.12

**Table 4:** Training and test samples of configuration variance.

Target type	Training set	Test set
BMP2	233 (Sn_9563)	196 (Sn_9566)
		196 (Sn_c21)

BTR70	233 (Sn_c71)	196 (Sn_c71)

T72	232 (Sn_132)	195 (Sn_812)
		191 (Sn_s7)

**Table 5:** Comparison with other methods under configuration variance.

Method type	CRC	KNN	SRC	SVM	CNN
Average recognition rate (%)	95.53	92.32	94.15	93.98	94.28

**Table 6:** Training and test sets from different depression angles.

Class	Training		Test	
	Depression	Number of samples	Depression	Number of samples
2S1		299	30°	288
			45°	303

BDRM2	17°	298	30°	287
			303

ZSU23/4		299	30°	288
			45°	303

The article "Automatic Target Recognition of SAR Images Using Collaborative Representation" was retracted in 2023. Reasons: signs of a paper mill; compromised peer review; unreliable results or conclusions.

**Table 7:** Performances of different methods under large depression angle variance.

Method type	Average recognition rate (%)	
	30°	45°
CRC	97.96	72.65
KNN	95.12	64.48
SRC	96.15	69.12
SVM	95.24	67.56
CNN	96.38	68.09

## Data Availability

The dataset can be accessed upon request.
